# Icariin Reduces Dopaminergic Neuronal Loss and Microglia-Mediated Inflammation *in Vivo* and *in Vitro*

This article has been retracted.

**DOI:** 10.3389/fnmol.2017.00441

**Published:** 2018-01-09

**Authors:** Guo-Qing Wang, Dai-Di Li, Chun Huang, Di-Sheng Lu, Chao Zhang, Shao-Yu Zhou, Jie Liu, Feng Zhang

**Affiliations:** Joint International Research Laboratory of Ethnomedicine of Ministry of Education and Key Laboratory of Basic Pharmacology of Ministry of Education, Zunyi Medical University, Zunyi, China

**Keywords:** Parkinson’s disease, microglia, neuroinflammation, icariin, neuroprotection

## Abstract

Parkinson’s disease (PD) is one of the most common neurodegenerative diseases characterized with a gradual loss of midbrain substantia nigra (SN) dopamine (DA) neurons. An excessive evidence demonstrated that microglia-mediated inflammation might be involved in the pathogenesis of PD. Thus, inhibition of neuroinflammation might possess a promising potential for PD treatment. Icariin (ICA), a single active component extracted from the Herba Epimedii, presents amounts of pharmacological properties, such as anti-inflammation, anti-oxidant, and anti-aging. Recent studies show ICA produced neuroprotection against brain dysfunction. However, the mechanisms underlying ICA-exerted neuroprotection are fully illuminated. In the present study, two different neurotoxins of 6-hydroxydopamine (6-OHDA) and lipopolysaccharide (LPS)-induced rat midbrain DA neuronal damage were applied to investigate the neuroprotective effects of ICA. In addition, primary rat midbrain neuron-glia co-cultures were performed to explore the mechanisms underlying ICA-mediated DA neuroprotection. *In vitro* data showed that ICA protected DA neurons from LPS/6-OHDA-induced DA neuronal damage and inhibited microglia activation and pro-inflammatory factors production via the suppression of nuclear factor-κB (NF-κB) pathway activation. In animal results, ICA significantly reduced microglia activation and significantly attenuated LPS/6-OHDA-induced DA neuronal loss and subsequent animal behavior changes. Together, ICA could protect DA neurons against LPS- and 6-OHDA-induced neurotoxicity both *in vivo* and *in vitro.* These actions might be closely associated with the inhibition of microglia-mediated neuroinflammation.

## Introduction

Parkinson’s disease (PD) is one of the most common neurodegenerative disease and characterized by the progressive loss of dopamine (DA) neurons in midbrain substantia nigra (SN) and the consequent movement malfunction (Towns, 2017). Although the mechanisms that drive the gradual nature remain elusive, to date, a great amount of evidence has documented microglia-mediated neuroinflammation is implicated in PD (Block and Hong, 2007; McKenzie et al., 2017). Microglia, the resident immune cells in the central nervous system, present a series of changes in morphology and function after activated by an acute insult to the CNS (Gao et al., 2002; Gao and Hong, 2008). Upon activation by brain injury or inflammogen exposure, microglia produce and secrete a great deal of pro-inflammatory factors, such as interleukin (IL)-1β, tumor necrosis factor α (TNF-α) and nitric oxide (NO). The generation and accumulation of these inflammatory mediators could not only further regulate immune reactions, but also injure DA neurons. Thus, it was suggested that the damaged DA neurons and the activated microglia might create a vicious self-amplifying cycle eliciting the prolonged and uncontrolled inflammation that promotes the chronic progression of PD (Gao and Hong, 2008; Gao et al., 2011). Taken together, microglia-mediated dynamic modulation of this neuroinflammation might be a key event in the degradation of DA neurons and inhibition of microglia-exerted vicious cycle could become a promising therapeutic potential for PD (Qian et al., 2010).

Icariin (ICA), a flavonoid derived from Herba Epimedii, shows a battery range of pharmacological properties, such as anti-inflammation, anti-oxidant, and anti-aging (Li et al., 2016; Xiao et al., 2016). Recently, ICA-mediated neuroprotection attracts a growing attention. Pharmacokineticly, ICA could pass through the blood–brain barrier (BBB) (Li and Wang, 2008). Additionally, our previous study indicated that ICA improved spatial learning and memory abilities in lipopolysaccharide (LPS)-induced rat brain dysfunction through the inhibition of hippocampus IL-1β and cyclooxygenase-2 (COX-2) expressions (Guo et al., 2010). Accumulating evidence indicates that, in addition to the inhibition of the activated innate immune cells (including microglia)-producing TNF-α and IL-1β, there is a constant depression of nuclear factor-kappa B (NF-κB) signaling activation in the hippocampus by ICA (Liu et al., 2015). Thus, ICA plays a counter-regulatory role in an attempt to suppress the neuroinflammation.

In the present study, we report that ICA conferred DA neuroprotection against 6-OHDA and LPS-induced neurotoxicity both *in vivo* and *in vitro*. In addition, this neuroprotection might be closely related to the inhibition of microglia activation and the subsequent neuroinflammatory reactions. It is for the first time to elaborate ICA-mediated neuroprotection and the underlying mechanisms.

## Materials and Methods

### Reagents

Icariin (ICA, purity 98%) was bought from Nanjing Zelang Medical Technology, Co., Ltd. (Nanjing, China). 6-OHDA (CAS 28094157) was from Sigma Chemical, Co. (St. Louis, MO, United States). LPS (*Escherichia coli* strain O111:B4) was purchased from Calbiochem (San Diego, CA, United States). Anti-Tyrosine Hydroxylase (TH) antibody, Anti-CR3 complement receptor (OX-42), Anti-Iba1 antibody, Goat Anti-Mouse IgG H&L (TRITC), and Goat Anti-Rabbit IgG H&L (TRITC) were bought from Abcam (Cambridge, MA, United States). NF-κB signaling pathway antibodies were the products of Cell Signaling Technology (Beverly, MA, United States). Biotinylated secondary antibodies and vectastain avidin–biotin complex (ABC) kits were purchased from Vector Laboratories (Burlingame, CA, United States). ELISA kits were purchased from R&D Systems (Minneapolis, MN, United States). Griess reagent was obtained from Beyotime Biotechnology (Shanghai, China).

### Animals and Treatment

Male SD rats (200–250 g) were purchased from the Experimental Animal Centre in the Third Military Medical University (Chongqing, China; Specific-pathogen-free Grade II). Animal experiments were in strict accordance with the Chinese Guidelines of Animal Care and Welfare and this study was approved by the Animal Care and Use Committee in Zunyi Medical University (Zunyi, China). LPS (5 μg in 5 μl of sterile saline) was injected into the right side of rat midbrain SN with the coordinates 4.8 mm posterior to bregma, 1.7 mm lateral to the midline and 8.2 mm ventral to the skull surface (Zhang et al., 2010). 6-OHDA (8 μg in 5 μl of saline with 0.2% vitamin C) was injected into the right side of SN with the coordinates 5.2 mm posterior to bregma, 2.4 mm lateral to the midline and 8.0 mm ventral to the skull surface (Hou et al., 2014). Daily intragastric administration of ICA (10 and 20 mg/kg) for 7 and 14 consecutive days was given beginning 24 h before LPS and 6-OHDA injection, respectively. Then, rotarod test was performed from the 5th day of LPS treatment and the 10th day of 6-OHDA treatment. One day after last ICA treatment, rats were sacrificed and the brains were collected.

### Primary Rat Midbrain Neuron-Glia Co-culture

Primary neuron-glia co-culture was from the ventral midbrain tissues of embryonic day 14 rats (Zhang et al., 2006). The dissociated cells were seeded at 5 × 10^5^/well in 24-well plate (DMEM/F12 containing 10% FBS, 10% HS, 1 mM sodium pyruvate, 2 mM L-glutamine and 0.1 mM non-essential amino acids). The cultures were maintained within a humidified atmosphere of 5% CO_2_ and 95% air in maintenance medium at 37°C. Seven-day-old cell cultures were performed for ICA treatments followed by LPS (10 ng/ml)/6-OHDA (40 μM) application. At the treatment time, cultures were composed of 10% microglia, 50% astroglia, and 40% neurons (including 1% DA neurons) (Hu et al., 2012).

### BV2 Cell Line

The mouse microglia cell line-BV2 was bought from the Cell Culture Center in the Institute of Basic Medical Sciences of Chinese Academy of Medical Sciences and Peking Union Medical College. BV2 cells were cultured in DMEM/F-12 medium and maintained at 37°C in a humidified incubator with 5% CO_2_.

### Immunocytochemical Staining

Cells were fixed in paraformaldehyde permeabilized with Triton X-100 and blocked with goat serum. DA neurons were identified with an anti-tyrosine hydroxylase (TH) antibody and activated microglia were recognized with an anti-OX-42 antibody. For LPS/6-OHDA-induced DA neuronal damage, cultures were incubated at 4°C overnight with anti-TH (1:300) and OX-42 (1:300) antibodies, followed by incubation with biotinylated secondary antibody for 1 h and then color was developed by 3, 3′-diaminobenzidine. For the quantification of TH-positive neurons and OX-42-positive microglia, four representative areas per well of the 24-well plate were counted. On each condition, three wells were applied for cell counting.

### TNF-α, IL-1β, and Nitrite Assay

The IL-1β and TNF-α levels in the culture medium were detected by ELISA kits. The NO production was determined by measurement of the accumulated levels of nitrite in the culture medium with Griess reagent.

### Western Blot Analysis

For the whole cell lysates extraction, cultures were homogenized in RIPA lysis buffer. The lysates were incubated for 30 min on ice and then centrifuged at 12,000 × *g* for 15 min. The protein concentration was quantified by BCA kit. The equal amount of total protein was separated on 10% *Bis*-Tris Nu-PAGE gel and transferred to PVDF membranes. The membranes were blocked with non-fat milk and then incubated with the following primary antibodies: ionized calcium-binding adapter molecule-1 (Iba-1, 1:800), TH (1:500), phosphorylated-p65 (p-p65, 1:1000), p65 (1:1000), and β-actin (1:2000). The membranes were incubated in horseradish peroxidase (HRP)-conjugated secondary antibodies at 1:3000 dilution followed by the blots developed with the enhanced chemiluminescence reagent.

### Rotarod Test

Rotarod test, consisted of cylindrical arrangement of thin steel rods, was performed for the investigation of muscular coordination. In the train, the speed was at 10 cycles/min and the cut-off time was 180 s (Khuwaja et al., 2011). Before the test start, all animals were trained on the rotarod till they stayed on it at least for the cut-off time. Rats were allowed to keep stationary for a while at 0 rpm and the rotational speed was gradually increased to 10 rpm in 20 s-interval till rats fell off from the rungs. Rat behavior changes were detected by two investigators and the mean duration time on the device was recorded (Hamm, 2001).

### DA Neuronal Counting in SN

Rat brain was cut into 35 μm transverse free-floating sections on a horizontal sliding microtome. Total 36 consecutive brain slices throughout the SN was collected. Every 6th section of a series of 36 consecutive brain slices was used to perform the immunocytochemical analysis. For LPS-induced DA neuronal damage, double-label immunofluorescence was employed with anti-OX-42 (1:500) antibodies and anti-TH antibodies (1:500), followed by incubation with FITC-conjugated goat anti-rabbit antibody (green) and anti-mouse antibody (red) secondary antibodies (1:1500). For 6-OHDA-induced DA neuronal damage, brain slices were immunostained with anti-OX-42 (1:300) antibodies and anti-TH antibodies (1:300), followed by incubation with biotinylated secondary antibody for 1 h. Digital images of SN TH-positive neurons and OX-42-positive microglia were obtained by an Olympus microscope (Olympus, Tokyo, Japan). DA neurotoxicity was evaluated by the quantification of TH-positive neuronal number and microglial activation was detected by the densitometry analysis of OX-42-positive microglia.

### Statistical Analysis

Data were presented as mean ± SEM. Statistical significance was analyzed by two-way ANOVA via GraphPad Prism software (GraphPad Software, Inc., San Diego, CA, United States). When ANOVA demonstrated the statistically significant differences, all pairwise comparisons among means were accessed by Bonferroni’s *post hoc t*-test with correction. A value of *p* < 0.05 or *p* < 0.01 was considered statistically significant.

## Results

### ICA Protected DA Neurons from LPS/6-OHDA-Elicited Neurotoxicity *in Vitro*

Primary rat midbrain neuron-glia co-cultures were treated with ICA (0.01 and 0.1 μM) for 30 min followed by LPS (10 ng/ml) or 6-OHDA (40 μM) application. Seven days later, LPS/6-OHDA-elicited DA neuronal damage was quantified by DA neuronal counting via immunocytochemical staining and TH protein expression through western blot assay. TH-positive neuronal counting detection indicated that LPS significantly decreased DA neuronal number and ICA ameliorated LPS-elicited DA neuronal injury (**Figures 1A,B**). Western blotting also indicated ICA attenuated LPS-elicited decrease of TH protein expression shown in **Figure 1C** and **Supplementary Figure S1A**. In 6-OHDA-treated neuron-glia co-cultures shown in **Figure 2**, 6-OHDA-induced reduction of DA neurons (**Figures 2A,B**) and decrease of TH protein expression (**Figure 2C** and **Supplementary Figure S1B**) was attenuated by ICA treatment.

**FIGURE 1:** Icariin (ICA) protected DA neurons against LPS-induced neurotoxicity *in vitro*. Rat primary midbrain neuron-glia cultures were pretreated with ICA (0.01 and 0.1 μM) for 30 min before LPS (10 ng/ml) treatment. Seven days later, ICA-produced neuroprotection was analyzed by the immunocytochemical analysis **(A)** and TH-positive neuron counting **(B)**. Representative images of immunostaining from three individual experiments were shown. Scale bar: 100 μm. The level of TH protein expression in the neuron-glia co-cultures was detected via western blot assay **(C)**. The ratio of densitometry values of TH with β-actin was assessed and normalized to each respective control group. Results were the mean ± SEM from three independent experiments performed in triplicate. ^∗^*p* < 0.05 or ^∗∗^*p* < 0.01 compared with the control cultures; ^#^*p* < 0.05 or ^##^*p* < 0.01 compared with LPS-treated cultures.

**FIGURE 2:** Icariin protected DA neurons against 6-OHDA-induced neurotoxicity *in vitro*. Rat primary midbrain neuron-glia cultures we re pretreated with ICA (0.01 and 0.1 μM) for 30 min before the treatment of 6-OHDA (40 μM). Seven days later, ICA-elicited neuroprotection was quantified by TH-positive neuron counting **(B)** through the immunocytochemical analysis. Representative images of immunostaining from three individual experiments were shown **(A)**. Scale bar: 100 μm. The level of TH protein expression in the neuron-glia cultures was measured with western blot analysis **(C)**. The ratio of densitometry values of TH with β-actin was assessed and normalized to each respective control group. Results were the mean ± SEM from three independent experiments performed in triplicate. ^∗^*p* < 0.05 compared with the control cultures; ^#^*p* < 0.05 compared with 6-OHDA-treated cultures.

### ICA Ameliorated LPS/6-OHDA-Elicited Microglia Activation *in Vitro*

Primary midbrain neuron-glia cultures were pretreated with ICA (0.01 and 0.1 μM) for 30 min and then stimulated by LPS/6-OHDA. Seven days later, the LPS/6-OHDA-induced microglia activation was analyzed by immunostaining with an anti-OX-42 (a marker of activated microglia used for immunostaining) antibody and western blot assay with an anti-Iba-1 (a marker of microglia including resting microglia and activated microglia) antibody. As shown in **Figures 3A,B**, LPS significantly induced microglia activation. However, ICA significantly attenuated LPS-induced microglia activation. In addition, to further investigate the inhibitory actions of ICA on LPS-elicited microglia activation, the whole cell lysis was collected and the effects of ICA on the protein expression of Iba-1 were determined. As shown in **Figure 3C** and **Supplementary Figure S1C**, LPS increased Iba-1 protein expression. However, ICA decreased LPS-induced Iba-1 protein expression. Moreover, in the neuron-glia co-cultures treated by 6-OHDA, more activated microglia were shown in 6-OHDA-treated cultures compared with the control cultures and ICA ameliorated 6-OHDA-induced microglia activation shown in **Figures 4A,B**. Furtherly, ICA inhibited 6-OHDA-induced increase of Iba-1 protein expression indicated in **Figure 4C** and **Supplementary Figure S1D**.

**FIGURE 3:** Icariin ameliorated LPS-induced microglial activation *in vitro.* Rat primary midbrain neuron-glia cultures were treated with ICA (0.01 and 0.1 μM) for 30 min and then stimulated by LPS (10 ng/ml). Seven days later, the activated microglia were detected by immunocytochemical staining with anti-OX-42 antibody. Representative images of immunostaining from three experiments were indicated **(A)**. Scale bar: 100 μm. The quantification of OX-42-positive microglia was performed **(B)**. The level of Iba1 protein expression in the neuron-glia co-cultures was detected via western blot assay **(C)**. The ratio of densitometry values of Iba1 with β-actin was assessed and normalized to each respective control group. Results were the mean ± SEM from three independent experiments performed in triplicate. ^∗^*p* < 0.05 compared with the control cultures; ^#^*p* < 0.05 compared with LPS-treated cultures.

**FIGURE 4:** Icariin attenuated 6-OHDA-induced microglial activation *in vitro*. Primary neuron-glia cultures were treated with ICA (0.01 and 0.1 μM) for 30 min followed by 6-OHDA (40 μM) treatment. Seven days later, the activated microglia were analyzed by immunocytochemical staining with an anti-OX-42 antibody. Representative images of immunostaining from three individual experiments were indicated **(A)**. Scale bar: 100 μm. The number of OX-42-positive microglia was counted **(B)**. The level of Iba1 protein expression in the neuron-glia cultures was quantified by western blot analysis **(C)**. The ratio of densitometry values of Iba1 with β-actin was assessed and normalized to each respective control group. Results were the mean ± SEM from three independent experiments performed in triplicate. ^∗^*p* < 0.05 compared with the control cultures; ^#^*p* < 0.05 or ^##^*p* < 0.01 compared with 6-OHDA-treated cultures.

### ICA Inhibited LPS/6-OHDA-Induced Release of Pro-inflammatory Factors *in Vitro*

To assess the inhibitory ability of ICA on the production of microglial pro-inflammatory factors, neuron-glia co-cultures were treated with ICA (0.01 and 0.1 μM) for 30 min followed by LPS/6-OHDA treatment. Twenty-four hour later, the release of TNF-α, IL-1β, and NO in the culture supernatant was detected. As indicated in **Figure 5**, the levels of TNF-α, IL-1β, and NO were increased in LPS/6-OHDA cultures. Compared with LPS/6-OHDA cultures, ICA significantly reduced the production of these pro-inflammatory factors.

**FIGURE 5:** Icariin inhibited LPS-/6-OHDA-induced release of pro-inflammatory factors *in vitro*. Primary midbrain neuron-glia cultures were treated with ICA (0.01 and 0.1 μM) for 30 min followed by LPS **(A)** or 6-OHDA **(B)** treatment. Twenty-four h later, the release of TNF-α, IL-1β, and NO in the culture medium was detected by ELISA and Griess regent, respectively. Results were the mean ± SEM from three independent experiments performed in triplicate. ^∗^*p* < 0.05 compared with the control cultures; ^#^*p* < 0.05 compared with LPS-/6-OHDA treated cultures.

### ICA Suppressed LPS/6-OHDA-Induced NF-κB Pathway Activation

It is well-known NF-κB signaling pathway was involved in the modulation of neuroinflammatory responses. Next, the actions of ICA on LPS/6-OHDA-elicited NF-κB pathway activation were detected. In primary neuron-glia cultures, ICA inhibited 6-OHDA-induced p65 phosphorylation shown in **Figure 6A** and **Supplementary Figure S2**. In BV2 cell line, LPS-induced p65 phosphorylation was attenuated by ICA treatment shown in **Figure 6B**.

**FIGURE 6:** Icariin attenuated LPS-/6-OHDA-induced NF-κB signaling pathway activation *in vitro*. Primary neuron-glia cultures **(A)** and BV2 cell line **(B)** were treated with ICA for 30 min and then stimulated with 6-OHDA or LPS for 24 h. The protein expressions of phosphorylated p65 (p-p65) and p65 were investigated by western blot analysis. The ratio of densitometry values of p-p65 with total p65 was analyzed and normalized to each respective control group. Results were the mean ± SEM from three independent experiments performed in triplicate. ^∗^*p* < 0.05 compared with the control cultures; ^#^*p* < 0.05 compared with 6-OHDA/LPS-treated cultures.

### ICA Attenuated LPS/6-OHDA-Induced DA Neuronal Loss and Microglia Activation *in Vivo*

With ICA-mediated neuroprotection *in vitro* indicated, ICA-produced DA neuroprotection against LPS/6-OHDA-induced neurotoxicity *in vivo* was further investigated. In LPS-elicited DA neuronal damage shown in **Figures 7A,B**, LPS significantly decreased the DA neurons in the SN and ICA ameliorated LPS-induced decrease of DA neuronal number. In parallel with DA neuronal loss, LPS induced microglia activation and this activated state of microglia was attenuated by ICA treatment shown in **Figure 7C**. In addition to DA neuronal number detection, rat behavior changes were also determined. As shown in **Figure 7D**, ICA attenuated LPS-induced decrease of the time stayed on the rod. In 6-OHDA-induced DA lesion shown in **Figure 8**, ICA improved 6-OHDA-induced decrease of DA neurons and activation of microglia in SN. These results were consistent with ICA-mediated neuroprotection against LPS-induced DA neurotoxicity.

**FIGURE 7:** Icariin attenuated LPS-Induced DA neuronal loss and microglial activation *in vivo*. Rats were given a single intranigral injection of LPS into the SN pars compacta on one side of rat brain followed by daily intragastric administration of ICA for 7 consecutive days. Then, rats were sacrificed and the brains were collected. Double-label immunofluorescence was performed by staining with anti-TH and anti-OX-42 antibodies (green fluorescence represented DA neurons and red fluorescence represented microglia) **(A)**. The “ellipse” presented the area of SN. Scale bar: 200 μm. The number of SN TH-positive neurons (mm^2^) was counted **(B)** and the quantification of SN OX-42-positive microglia number was performed **(C)**. Rat behavior changes were analyzed through rotarod test. The time stayed in rod was recorded **(D)**. Results were the mean ± SEM from six rats (*n* = 6). ^∗^*p* < 0.05 or ^∗∗^*p* < 0.01 compared with the control group; ^#^*p* < 0.05 or ^##^*p* < 0.01 compared with LPS-treated group.

**FIGURE 8:** Icariin alleviated 6-OHDA-induced DA neuronal impairment and microglial activation *in vivo*. After daily intragastric treatment of ICA for 14 consecutive days, rats were sacrificed and the brains sections were immunostained with anti-TH antibody **(A)**. The number of TH-positive neurons in the SN was counted **(B)**. Microglia activation in SN was assessed by immunostaining with anti-OX-42 antibody **(C)**. The densitometry analysis of SN OX-42-positive microglia was analyzed **(D)**. The “ellipse” presented the area of SN. Scale bar: 200 μm. In order to verify the effects of 6-OHDA on muscle coordination, the time stayed in rod was tested beginning 10th day after 6-OHDA injection **(E)**. Results were the mean ± SEM from six rats (*n* = 6). ^∗^*p* < 0.05 or ^∗∗^*p* < 0.01 compared with the control group; ^#^*p* < 0.05 or ^##^*p* < 0.01 compared with LPS-treated group.

## Discussion

The present study presented that ICA conferred significant DA neuroprotection against 6-OHDA/LPS-induced neurotoxicity and inhibited microglia activation and the pro-inflammatory factors release. In *in vitro* studies, ICA protected DA neurons from LPS/6-OHDA-induced DA neuronal damage and reduced microglia activation and pro-inflammatory factors production via the suppression of NF-κB pathway activation. In animal studies, ICA significantly reduced microglia activation and significantly attenuated LPS/6-OHDA- induced DA neuronal loss and subsequent animal behavior changes. These findings suggest that ICA might hold the promising therapeutic properties on PD.

Several lines of evidence confirm that neuroinflammation was closely involved in the pathogenesis of PD. As the brain resident immune cells, microglia play a pivotal role in the neuroinflammation. In response to brain injury or immunological challenges, microglia release various kinds of pro-inflammatory and cytotoxic factors. The accumulation of these factors further resulted in the progressive loss of DA neurons. It was interesting to note that ICA produced neuroprotection against DA neurotoxicity induced by LPS and 6-OHDA, two toxins with different modes of functions (Badshah et al., 2016; Wasik et al., 2016). 6-OHDA was a hydroxyl derivative of DA and competed for DA uptake sites and undergoes auto-oxidation, leading to direct DA neuronal damage by producing neurotoxic substances (Im et al., 2016; Song et al., 2016). However, the continuing damaged DA neurons also produce various types of neurotoxic soluble factors, such as α-synuclein and damage-associated molecular patterns (DAMPs), which in turn caused microglia activation. LPS was a potent inflammatory substance and directly induced microglia activation-mediated neuroinflammation and then the activated microglia further caused DA neuronal damage (Fantoni et al., 2017). Unlike LPS-elicited direct microglia activation, 6-OHDA led to the selective DA neuronal dysfunction/death and secondary the activation of microglia (Liu and Bing, 2011). Either kind of microglia activation elicited by LPS and 6-OHDA might further damage DA neurons in a “self-propelling” vicious cycle and finally result in the progression of DA neurodegeneration. In this study, both 6-OHDA and LPS caused DA neuronal loss and microglia activation. However, ICA seemed to protect DA neurons through the inhibition of microglia activation and thus halt this vicious cycle running. In addition, tt is well-known that the pathological hallmark of PD is the formation of α-synuclein-containing Lewy Body in midbrain dopaminergic neurons. Thus, it is quite interesting to investigate the effects of ICA on the contents of α-synuclein in dopaminergic neurons. Since LPS and 6-OHDA are two acute toxins to induce dopaminergic neuronal damage, no significant α-synuclein accumulation was discerned. Thus, to explore the effects of ICA on other PD animal models, such as overexpressing human A53T mutant α-synuclein animal model, warrants further elucidation.

Numerous studies have suggested that microglial pro-inflammatory and cytotoxic factors, such as IL-1β, NO and TNF-α, were recognized to contribute to DA neurodegeneration (Choi et al., 2009). Therefore, reduction of neuroinflammatory factors production might present a promising therapeutic potential for PD. In LPS-treated neuron-glia co-cultures, a significant increase of pro-inflammatory factors production in LPS group and ICA obviously inhibited LPS-induced release of these factors. Furthermore, in 6-OHDA-treated co-cultures, an increased production of pro-inflammatory factors was shown in 6-OHDA group. This exactly suggested that 6-OHDA directly damaged DA neurons and the injured DA neurons excreted various neurotoxic factors and these factors further induced microglia activation and then these activated microglia produced amounts of pro-inflammatory factors. However, ICA still ameliorated 6-OHDA-induced microglial pro-inflammatory factors production.

Promoter regions of pro-inflammatory factors contained the DNA binding site of NF-κB. In addition, suppression of NF-κB activation reduced the pro-inflammatory factors release. Also, NF-κB activation was discerned within PD patients SN and PD animal model (Hunot et al., 1997; Ghosh et al., 2007). These results strongly suggest NF-κB was the key regulator of neuroinflammation. In the resting conditions, NF-κB dimers (p50 and p65) were sequestered in cytosol via binding to its inhibitor, IκB. However, activation of NF-κB required the nuclear translocation of p50 and p65 following rapid IκB phosphorylation, degradation, and release (Zhang and Ghosh, 2001). Furtherly, selective suppression of NF-κB activation attenuated microglia activation and protected from DA neuronal loss (Ghosh et al., 2007). Furthermore, inhibition of NF-κB activation and the subsequent pro-inflammatory factors production participated in the neuroprotection against LPS-induced DA neurotoxicity (Xing et al., 2007). In this study, we employed two different cell cultures, primary neuron-glia co-cultures and BV2 cell line, to verify whether ICA inhibited microglial pro-inflammatory factors production via the inhibition of NF-κB activation. Here, LPS and 6-OHDA induced NF-κB activation in these two cell cultures and ICA alleviated LPS/6-OHDA-induced NF-κB activation.

So far, no effective therapy is available to stop PD progression. Although, the dopamine agonist or levo-dopa is the standard treatment for PD, it is frequently associated with a series of side effects and unsatisfactory outcomes. Thus, to understand the mechanisms underlying PD process and develop the effective therapeutic approaches to halt the progression of PD is of paramount significance. Since neuroinflammation is verified to an important contributor to the acceleration of PD progression, this process may be an important breakpoint for the disease control. Thus, treatment with anti-inflammatory agents is gaining higher importance on PD therapy. The present study demonstrated that ICA could afford neuroprotection against LPS-/6-OHDA-induced DA neurotoxicity both *in vivo* and *in vitro* by inhibiting microglial activation (**Supplementary Figure S3**). Although this apparently promising perspective for future application of ICA potential treatment for PD, most of the findings resulted from experimental animal models and thus need be rigorously confirmed in the human studies.

## Conclusion

This study illustrates that ICA could protect DA neurons against LPS- and 6-OHDA-induced neurotoxicity both *in vivo* and *in vitro.* These actions might be closely associated with the inhibition of microglia-mediated neuroinflammation.

## Author Contributions

FZ conceived and designed all the experiments. G-QW, D-DL, CH, D-SL, and CZ performed the experiments. FZ, S-YZ, and JL finished the data analysis. FZ, G-QW, D-DL, and CH wrote and revised the manuscript. All the authors reviewed the manuscript and approved the submitted manuscript.

## Conflict of Interest Statement

The authors declare that the research was conducted in the absence of any commercial or financial relationships that could be construed as a potential conflict of interest.

## Supplementary Material

FIGURE S1 Icariin attenuated dopaminergic neuronal loss and microglia activation. Effects of Icariin on TH protein expression after LPS **(A)** and 6-OHDA **(B)** treatment were detected. Effects of Icariin on Iba1 protein expression induced by LPS **(C)** and 6-OHDA **(D)** application were measured.

FIGURE S2 Icariin ameliorated p65 phosphorylation induced by LPS and 6-OHDA.

FIGURE S2 Icariin reduced dopaminergic neuronal loss and microglia-mediated inflammation.
